# Feasibility Analysis and Discrete Dynamic Modeling of Physical Education Teaching Strategy Based on Intelligent Computing

**DOI:** 10.1155/2022/4093924

**Published:** 2022-06-07

**Authors:** Ge Wang

**Affiliations:** School of Physical Education and Sport Science, Fujian Normal University, 350117 Fuzhou, Fujian, China

## Abstract

With the advent of the information age, computer technology is also widely used in various fields. In the field of education, physical education teaching strategy has always been the focus of many educators. In order to optimize physical education teaching strategies and improve teaching quality, this paper proposes a new intelligent computing technology. This technology has excellent innovation in the engineering design field of physical education teaching strategy reform and innovation and combines Intelligent Computing with physical education teaching strategy to explore the feasibility and effectiveness of physical education teaching strategy reform and innovation. On the basis of intelligent computing algorithm, this paper analyzes the visualization strategy scheme brought by intelligent computing classroom to physical education teaching. This paper analyzes the feasibility of students' feedback after the reform of the physical education teaching strategy. Finally, the big data discrete dynamic modeling technology is used to dynamically model and analyze the students' learning behavior and effect after the reform and innovation of physical education teaching strategy. Combined with the analysis data and students' behavior feedback, this paper analyzes the feasibility of the physical education teaching strategy after the reform and innovation. The results show that the visualization scheme of physical education teaching strategy based on intelligent computing can help students understand theoretical knowledge and realize the transformation from static classroom to dynamic classroom. It enhances students' practical activities and perceptual knowledge and is of great help to students' physical education learning effect. In the discrete dynamic modeling analysis, the feasibility of physical education teaching strategy reform is very important.

## 1. Introduction

With the influence of examination-oriented education in China, the decline in students' physical quality in China is very serious (Wan et al. 2021) [1]. There are many diseases such as myopia, obesity, and weakness. Good physical education teaching can help students improve this situation. Therefore, the task of physical education teaching strategy reform in China is imminent (Jennina et al. 2021) [2]. Comprehensively improving students' physical quality and physical education achievements has become one of the teaching objectives of each university. More and more colleges and universities begin to pay attention to the reform of students' physical education teaching strategies. However, there are still many deficiencies in the actual process of teaching strategy reform and innovation. As a result, students cannot give full play to their strengths and form good learning habits in sports activities (Hao et al. 2021) [3]. Among them, the factors affecting the reform of physical education teaching strategies include the low attention of schools. In carrying out sports activities, many colleges and universities do not pay enough attention to the impact of teaching itself (Yuchen et al. 2021) [4]. Physical education teaching is not only to improve students' physical performance but also to improve students' physical quality and comprehensive quality. Students need to improve their physical environment through physical education and physical exercise. Moreover, in school social communication, a good physical education teaching environment can help students change the introversion trend and expand communicative activities (Li et al. 2021) [5].

Most teachers only regard physical education courses as free activity time in physical education teaching, without clear teaching objectives (Liu et al. 2021) [6]. In the actual teaching process, I did not understand how to highlight the characteristics of sports and training direction. Teachers lack the combination of the theoretical basis and teaching activities, resulting in students' interest in sports cannot be effectively improved (Yang et al. 2021) [7]. The teaching mode of many colleges and universities is relatively backward, and the traditional physical education teaching method still exists in many schools. Teachers' teaching to students is mainly theoretical learning, supplemented by physical training [8]. This traditional teaching mode has a great impact on students' physical education development. In the learning process, it does not reflect that students are the main body of learning and lack of subjective initiative. With the combination of education and information technology, more and more physical education teaching strategies began to appear and achieved good results and teaching results (Lin et al. 2021) [9]. As a modern auxiliary teaching tool, intelligent computing can bring new opportunities for the physical education teaching environment. This method was originally used in the field of engineering and can simulate biological mechanism and evolution process with the help of a computer. It provides technical support for information acquisition and information processing. It has achieved good results in the fields of virtual modeling, image recognition, image processing, information processing, prediction analysis, and so on. Facing the single form of traditional physical education teaching strategy, this paper combines intelligent computing with physical education teaching to explore the reform, innovation, and feasibility analysis of teaching strategy.

Optimizing physical education teaching strategies and improving teaching quality are the main contents of the reform and innovation of physical education teaching strategies, including implementing the guiding principle of health first in teaching guiding ideology. In the relationship between teaching and learning, it emphasizes the equality between teachers and students, cooperation, and interaction, and students are the main body of teaching. In the concept structure of teaching, it emphasizes that teaching activities are the organic unity of three psychological activities: cognition, emotion, and behavior. Teaching design should create conditions for students' independent choice and active exploration in the teaching process, advocate teaching democracy, make students' learning an active and personalized process under the guidance of teachers, and emphasize the formation of students' self-study ability.

This paper is mainly divided into three parts. The first part is a basic understanding of the reform and innovation of physical education teaching strategies and puts forward the teaching strategies and teaching modes of intelligent computing. The research status of discrete dynamic modeling technology used in feasibility analysis is analyzed. The second part first studies the mode of Intelligent Computing physical education teaching strategy and analyzes the application of intelligent computing algorithm in the feasibility study. This paper studies the changes in students' behavior after the reform of the Intelligent Computing physical education teaching strategy. Finally, the discrete dynamic modeling technology is used to analyze the feasibility of physical education teaching strategy reform and innovation. The third part analyzes the teaching environment after the reform of the physical education teaching strategy and the results of the feasibility study of the Intelligent Computing teaching mode.

## 2. Related Work

The reform of the physical education teaching strategy is a complex process and structure. Not only do schools need to pay more attention to physical education but also students need to form a good physical education classroom atmosphere (Liao et al. 2021) [10]. In the physical education teaching environment, teachers should give full play to their professional skills, analyze students' physical and mental characteristics, and formulate targeted teaching strategies (Bian et al. 2021) [11]. In the reform of physical education teaching strategy, we first need to solve the importance of this industry, make use of its own advantages to spread and influence in various aspects, improve people's understanding of sports, and use their spare time to help students take physical exercise. In the reform of teaching strategies, it needs to be formulated according to the physical and mental characteristics of students, and the time of sports activities cannot be reduced in order to meet the needs of examination-oriented education (Zhang et al. 2021) [12]. We use the characteristics of intelligent computing to improve physical education teaching strategies in order to explore the feasibility of this method. This paper uses big data discrete dynamic modeling technology to analyze the feasibility. Discrete dynamic modeling technology can quickly deal with the problem of excessive data in big data environment, which provides effective help for system operation and efficiency improvement. In the feasibility analysis, combined with the changes in students' own behavior, we study the dynamic changes before and after the improvement of the Intelligent Computing physical education teaching strategy. Finally, it provides accurate data sources for exploring the feasibility of teaching strategy reform and innovation. Next, we will briefly describe the application status of big data discrete dynamic modeling technology in various countries.

Japan does not pay much attention to the ecological environment. Therefore, with the progress and development of the times, they mainly study the protection and utilization of sustainable energy and renewable energy (Lin et al. 2021) [13]. Wind power generation has always been a large model in renewable energy. With the continuous bad changes in the ecological environment, they pay more attention to the research on the operation process of wind power generation. Wind turbines are prone to damage during operation. In order to effectively monitor the aging degree of components, they apply discrete dynamic modeling technology here to timely grasp the operation state of the motor and ensure stable operation.

Enterprise development in Korea has always been the main source of the national economy. With the popularization of the Internet, the information system has also changed (Guan et al. 2021) [14]. Enterprises have been slow to use and accept big data. In order to improve this situation, they use big data technology to optimize and dynamically model enterprise management. Mainly combined with various factors affecting the enterprise environment, this paper constructs a dynamic model of data analysis and processing and finally realizes the purpose of optimizing the enterprise development process.

The United States is relatively advanced in the development of the military field. Their military strength is very strong, but computer technology is also a field that cannot be underestimated [15]. They have provided many effective achievements and research in the development of information technology. Military equipment operation system usually has minor faults, which is not conducive to their national security and guarantee. Therefore, they use big data technology to dynamically model and analyze the data source of equipment operation and build a prediction model to give early warning of possible fault factors in the system. Thus, the purpose of reducing maintenance cost and overhaul cost is realized. Based on the development status of discrete dynamic modeling technology in various countries, this paper studies the feasibility analysis of Intelligent Computing physical education teaching strategy reform.

## 3. Methodology

### 3.1. Feasibility Study on the Reform and Innovation of Physical Education Teaching Strategy Based on Intelligent Computing

At this stage, most teaching methods in physical education teaching strategies have undergone basic reform and innovation. Traditional teaching mode and innovative teaching mode are parallel to each other. Most colleges and universities adopt traditional teaching, optional physical education, and free activity teaching. Through literature survey, we know that ordinary teaching methods have been relatively rare. The current physical education teaching mode has been basically improved in combination with modern educational technology. Traditional teaching strategies only appear in track and field, shot put, gymnastics, and other events. The physical education curriculum in most colleges and universities is also relatively single, and practical knowledge and teaching mode are relatively rare. This situation leads to the fact that the physical education curriculum in colleges and universities does not have its own characteristics and cannot attract students to study and stimulate interest. In the teaching strategy of intelligent computing, we use the efficient computer language program MATLAB as the core technology of visual teaching. It can process a large amount of data and information and realize analysis and sorting. It provides technical support in visual physical education teaching strategy. Visual teaching in physical education teaching strategy refers to the concretization of abstract actions by using simulation technology. In sports training, the most common observation methods are video observation and three-dimensional dynamic photography, which are established on the basis of science. Human motion simulation technology mainly includes the establishment of the human model, the collection of more real physical reaction signals of the human body under specific conditions, the process of computer simulating human real motion, and so on. This technology is a major breakthrough of information technology in the process of sports. It can promote the development of sports and the development of three-dimensional dynamic simulation technology in sports, analyze and extract the theoretical knowledge from the essence, and show it intuitively. In traditional teaching, in addition to using body language to convey information, students can also perceive actions in virtual simulation. We apply MATLAB visualization technology to the teaching strategy of sports intelligent computing, which can enhance students' sensory understanding. In the process of studying the reform of Intelligent Computing physical education teaching strategy, it is necessary to complete three parts: theory teaching, actionability, and curriculum practice. We need to maximize the improvement of the physical education curriculum in a limited time. Compared with ordinary courses, this model has a shorter teaching time. In the reform and innovation of physical education teaching strategies, we need to pay more attention to students' thinking divergence ability and practical ability. Different from the traditional classroom, the optimized classroom can enrich students' ability to acquire knowledge. In Intelligent Computing physical education teaching, theory and practice need to be highly integrated. The traditional physical education teaching strategy only pays attention to the academic achievement and actual effect but does not pay attention to the teaching process. With the continuous development of educational ideas, in the process of education, we no longer only pay attention to the teaching of relevant knowledge and skills. At the same time, we also need to pay more attention to the awakening of students' self-spirit and constantly stimulate students' thinking of self-thinking and self-creation. When this phenomenon is fed back to the computer industry and artificial intelligence teaching, it is necessary to cultivate computing thinking in the process of basic computer knowledge teaching and skill training. Of course, due to the influence of traditional educational thought, the cultivation of computing thinking is relatively weak. However, intelligent computing course needs to cultivate students to combine theory with practice and be able to deal with technical problems by themselves. This cross-teaching strategy mode is shown in Figure 1.

As can be seen from Figure 1, this physical education teaching strategy includes theoretical teaching and innovation as well as practical exercises. It fully reflects the innovation and reform effect of teaching strategies and has a positive impact on students' physical education teaching activities. In order to explore the feasibility of physical education teaching strategy reform and innovation, we need huge data as the basis of analysis results. In dealing with massive data, intelligent computing algorithm can improve the running speed of the system on the premise of ensuring real time. Firstly, the feasibility analysis model is established, and the test values of data accuracy are as follows:

(1) $$\begin{array}{c} M_{t+1}=M_{t}+w\left(m_{t}-M_{t}\right), \end{array}$$

where *M*_*t*_is the prediction data at each time and *w* is the weight coefficient. Set that the changes between adjacent data are equal, and the calculation formula is

(2) $$\begin{array}{c} \varepsilon =M_{t}-M_{k-1}. \end{array}$$

In order to solve the error coefficient in data calculation, we will test the multiple prediction results in the way of average:

(3) $$\begin{array}{c} M=\frac{\sum_{K=1}^{n}M_{K}}{n}. \end{array}$$

Judge the difference between the two coefficients to illustrate the changing trend of error rate when the current data increase with the number. In order to deal with high-dimensional data sets and prevent the fitting phenomenon, we need to classify and balance the data samples, increase the fault tolerance of the algorithm, and set the calculation formula of the sample characteristic index as follows:

(4) $$\begin{array}{c} G_{m}=\sum_{k=1}^{\left|k\right|}\sum_{k\neq k}\text{pmkpmk}{\;}^{\prime }=1-\sum_{k=1}^{\left|k\right|}p^{2}\text{mk}. \end{array}$$

In the formula, *k* represents the sample category and pmk represents the proportion of nodes and coefficients. Secondly, the importance of the eigenvector in the calculation node is expressed as follows:

(5) $$\begin{array}{c} {\text{VIM}}_{\text{jm}}^{\left(\text{Gini}\right)}=G_{m}-G_{i}-G_{r}. \end{array}$$

In the formula, *G*_*i*_ and *G*_*r*_, respectively, represent the relationship index in the node. If the eigenvalue is in the set state, the weight is

(6) $$\begin{array}{c} {\text{VIM}}_{\text{jm}}^{\left(\text{Gini}\right)}=\sum_{mɛM}{\text{VIM}}_{im}^{\left(\text{Gini}\right)}. \end{array}$$

Assuming that there are multiple parent nodes in the algorithm, the formula is defined as follows when calculating the feasibility of characteristic data

(7) $$\begin{array}{c} {\text{VIM}}_{i}^{\left(\text{Gini}\right)}=\sum_{j=1}^{n}{\text{VIM}}_{ji}^{\left(\text{Gini}\right)}. \end{array}$$

Finally, the calculated feasibility score is summarized by normalization as follows:

(8) $$\begin{array}{c} {\text{VIM}}_{i}=\frac{{\text{VIM}}_{i}}{\sum_{j=1}^{m}{\text{VIM}}_{j}}. \end{array}$$

To sum up, the calculation can obtain the feasibility data of the reform model of physical education teaching strategy and provide accurate data support for the reform process of physical education teaching strategy. We summarize the flow of the intelligent computing model as shown in Figure 2.

As can be seen from Figure 2, first initialize the calculation parameters of the algorithm and arrange the factors affecting the data results. Finally, according to the adaptability of each data, the data are divided and processed uniformly. According to the feasibility results of physical education teaching strategy reform and innovation, the optimized physical education teaching model is more suitable for students' physical activities. The visual teaching of intelligent computing can also optimize the teaching according to the concept of combining theory with practice. With its own advantages of image, vividness, and intuition, visual teaching arranges a large amount of theoretical information into a collection. It is convenient for teachers to summarize teaching priorities and help students show their thinking through practical activities in combination with theoretical knowledge.

### 3.2. Feasibility Study on the Reform and Innovation of Physical Education Teaching Strategy Based on Discrete Dynamic Modeling Analysis

With the advent of the information age, information-based teaching mode and intelligent teaching mode have been gradually applied in the field of education. With the increasing demand for learning, it is necessary to study the theoretical knowledge that cannot be expressed by action in physical education teaching. We began to explore the practical application of information-based teaching methods in physical education. Intelligent computing visual physical education teaching strategy can make physical education technology and action clearly displayed in front of students. In traditional physical education teaching strategies, teachers can only teach movements through multiple demonstrations. This model is no longer applicable to today's environment. Therefore, a series of reforms and innovations have been carried out for physical education teaching strategies. In order to better explore the feasibility of reform and innovation, this paper uses big data discrete dynamic modeling technology to analyze the behavior of physical education learners. Because the work task and processing speed of the database in the big data environment are the main factors affecting the result judgment, the traditional data processing technology cannot face this dynamic and complex environment, so it is necessary to use discrete dynamic modeling to process the data set. In the selection of hardware system, make full use of the modern platform and combine the prediction model with historical experience to make the data processing model more intelligent. Be able to adapt to the changes in dynamic data and work content. Firstly, we reduce the error rate of data results based on Bayesian theory. The behavior of physical education learners is regarded as a feature vector. The eigenvalues are expressed by conditional coefficients. Define the main behavior of data in different categories and different sample characteristics, then

(9) $$\begin{array}{c} P\left(C_{i}|X\right)=\frac{P\left(X|C_{i}\right)P\left(C_{i}\right)}{P\left(X\right)}. \end{array}$$

The assumed independence of the above formula is

(10) $$\begin{array}{c} P\left(X|C_{i}\right)=\overset{M}{\underset{j=1}{∐}}P\left(X_{i}|C_{i}\right). \end{array}$$

According to the above formula, we can divide the data processing into three parts. The first part is data mining and sorting, the second part is data visualization calculation, and the third part is to ensure the accuracy and independence of calculation. In learner behavior analysis, the correct rate and error rate of each behavior are different. A sports project needs a variety of learning behaviors to carry out a feasibility analysis. We mark the nodes in the behavior. When the value of the teaching strategy is a fixed value, we can obtain the learners' learning state. If learners can master this sports skill in this teaching strategy, it can be expressed as

(11) $$\begin{array}{c} P\left(C_{n}=\text{false}|K_{n}=\text{true}\right),\\ P=\frac{\exp\left(-\sum_{j=1}^{n}\delta_{j}s_{j}^{n}+\gamma \right)}{1+\exp\left(-\sum_{j=1}^{n}\delta_{j}s_{j}^{n}+\gamma \right)}. \end{array}$$

In the formula, *P* represents learning efficiency and *K*_*n*_ represents accuracy.

If we cannot master this sports skill in learning, the coefficient of teaching strategy can be expressed by visual data. The calculation equation obtained by logarithmic regression expansion is

(12) $$\begin{array}{c} P\left(G_{n}\right)=P\left(C_{n}=\text{true}|K_{n}=\text{false}\right),\\ P\left(G_{n}\right)=\frac{1}{1+\exp\left(-\sum_{j=1}^{n}\alpha_{j}s_{j}^{n}+\beta \right)}. \end{array}$$

In the formula, *α*_*j*_ and *s*_*j*_^*n*^ can represent the factors affecting the correctness and error of feasibility judgment, and *β* is the calculated deviation. Finally, the learning probability and mastery degree are expressed by the following probability formula:

(13) $$\begin{array}{c} P\left(K_{n+1}\right)=\text{true}|=K_{n}=\text{false}=\frac{1}{1+\text{exp}\left(-\sum_{j=1}^{n}\alpha_{j}s_{n}^{\left(j\right)}+\beta \right)}. \end{array}$$

According to the above formula, we can get the feasibility analysis results of discrete dynamic modeling technology on the reform and innovation of physical education teaching strategies. The teaching effect is known through the judgment of learners' behavior correctness and the mastery of sports skills. We will analyze the students' learning effect before and after the reform of the physical education teaching strategy as shown in Figure 3.

It can be seen from Figure 3 that after the reform and innovation of physical education teaching strategies, most students can improve their mastery of physical education skills. It has been well applied in sports.

## 4. Result Analysis and Discussion

### 4.1. Analysis of Feasibility Study Results of Physical Education Teaching Strategy Reform and Innovation Based on Intelligent Computing

The core content of optimization in the reform and innovation of physical education teaching strategy lies in the teaching mode. In traditional physical education, teachers are the main body and students are the object of imitation. Under this mode, students' own enthusiasm and initiative have been restrained, and their understanding of sports is not deep enough. Teachers' professional level and teaching content can affect students' learning interest to a certain extent. In order to improve this situation, this paper combines the visual teaching design in Intelligent Computing with physical education and puts forward a dynamic and innovative teaching strategy. In order to study the feasibility of physical education teaching strategy reform, we need formal modeling and intelligent calculation of learner evaluation. In the evaluation of physical education teaching, we should emphasize the task of physical education teaching and skill development. In testing, actions are often separated. What students learn are specific skills, which are often practiced under the condition of decomposition. Then, use standardized tests to test their ability to do these decomposition skills. Traditional evaluation methods cannot meet the current needs. We need to dynamically observe students' state and learning performance in sports activities. This demand brings some difficulties to the feasibility evaluation and analysis. We use the intelligent calculation algorithm to analyze the error of the student evaluation coefficient and test whether the evaluation results meet the accuracy requirements, which can be helpful for feasibility judgment. Next, we compare the accuracy changes of data before and after intelligent computing as shown in Figure 4.

It can be seen from Figure 4 that the information data processed by intelligent computing can ensure a certain accuracy in a massive range. According to the evaluation results, we want to intervene students' physical education teaching strategies and determine whether the current interaction state of students meets the expected effect. According to the students' feedback, we know that the reform and innovation of physical education teaching strategies can have a positive impact on teaching activities. It has certain feasibility in the actual teaching effect.

### 4.2. Analysis of Feasibility Study Results of Physical Education Teaching Strategy Reform and Innovation Based on Discrete Dynamic Modeling Analysis

In the reform and innovation of physical education teaching strategies, we find that in order to mobilize students' interest in physical activities, this teaching model must be integrated with information skills, that is, integrated with auditory, tactile, and visual information to improve students' desire for exploration. The use of video or pictures in multimedia technology to explain sports movements separately is of great help to students' understanding and mastering skills. We found that after the reform and innovation of the physical education teaching strategy, it is very helpful for students to master knowledge points. Teachers only need to point out the wrong actions in training in time to help students exercise correctly. The traditional teaching strategy is only simple teaching according to the classroom form. Using the teaching strategy of information combination can make the physical education classroom more vivid in an intuitive and visual way. In the feasibility analysis of physical education teaching strategy reform and innovation, we use discrete dynamic modeling to predict and judge the results. Discrete dynamic modeling technology can quickly process a large amount of data information and ensure the accuracy of data. In terms of data feedback efficiency, discrete modeling technology also has good performance. We compare the feedback of the traditional prediction model with the discrete dynamic model as shown in Figure 5.

It can be seen from Figure 5 that the system model constructed by discrete dynamic modeling technology can stabilize the feedback efficiency when the data are increasing. Compared with the traditional prediction model, it has high applicability. In the reform and innovation of physical education teaching strategies, it can bring accurate judgment and rapid feedback to the calculation results. After feasibility analysis, we put forward some suggestions on the reform of the physical education teaching strategy. First, improve the teaching mode and set up physical education courses according to different types. For example, football, basketball, and yoga give full play to these professional advantages to the students. Let students drive students' learning and form a community model. Secondly, improving teaching facilities and sports environment can increase the atmosphere for students' sports activities. At the same time, it can ensure that students will not be injured due to sports conditions. Adding sports facilities can make students pay more attention to exercise. The last is to improve the level of teachers. A good physical education teaching strategy needs a qualified teacher to improve. PE teachers with professional and technical level can make students better understand sports activities and ensure the accuracy of posture in sports movement training.

## 5. Conclusion

With the improvement of the overall quality of the whole people, sports have become a necessary content in daily life. All colleges and universities have reformed and innovated the physical education teaching mode and strategy. Due to the defects of traditional physical education equipment and the influence of external factors, students' interest in physical activities is not high. Most students have poor physical quality in the examination-oriented education environment. More and more parents and teachers begin to pay attention to students' health. Therefore, it is imperative to reform and innovate physical education teaching strategies. The actual changes after the reform and innovation of physical education teaching strategies need further analysis and research. This paper analyzes the feasibility of physical education teaching strategy reform and innovation by using intelligent computing algorithm and big data discrete dynamic modeling technology. Firstly, according to the defects of physical education teaching strategies, this paper puts forward the ways and methods of reform and innovation. This paper briefly analyzes the application status of big data discrete dynamic modeling technology in various countries. Combining the traditional classroom with the teaching method of intelligent computing, the teaching effect is analyzed by using the intelligent computing model. Finally, we compare the behavior characteristics of students before and after the reform and innovation of physical education teaching strategies, conduct discrete dynamic modeling analysis, and integrate the data results of dynamic analysis with students' learning attitude and effect to achieve the purpose of feasibility analysis. The results show that the reform and innovation of physical education teaching strategies can help students improve physical exercise activities and lay a foundation for the growth of students' interest in sports and help teachers improve the bad situation of students' sports activities and realize the concept of teaching integration and students' physical and mental growth.

## Figures and Tables

**Figure 1:** Cross-teaching strategy model.

**Figure 2:** Process of intelligent computing model.

**Figure 3:** Analysis of students' learning effect before and after the reform of physical education teaching strategy.

**Figure 4:** Changes in data accuracy before and after Intelligent Computing.

**Figure 5:** Comparison between feedback of traditional prediction model and discrete dynamic model.

## Data Availability

The data used to support the findings of this study are included in the article.
